# The Use of Safflower (Carthamus tinctorius) in Treating Depression and Anxiety

**DOI:** 10.7759/cureus.22278

**Published:** 2022-02-16

**Authors:** Asma S Albaiz

**Affiliations:** 1 Psychiatry, Prince Sultan Military Medical City, Riyadh, SAU; 2 Psychiatry, Queen's University, Kingston, CAN

**Keywords:** psychological stress, anxiety, depression, carthamus tinctorius, safflower

## Abstract

Objective

In the era of evidence-based medicine, research in the area of herbal psychopharmacology has increased dramatically in recent decades. To date, however, there is no comprehensive review of safflower as an herbal antidepressant and anxiolytic with details on its psychopharmacology and applications in depression and anxiety.

Methods

This research is a review and qualitative research through an electronic survey among the Saudi population, thus assessing their knowledge about using safflower in treating depression and anxiety. The survey was distributed in Saudi Arabia in December 2021 and the results were finalized in January 2022.

Results

A total of 1074 Saudi participants were included in the study; 1002 (93.3%) participants reported knowing safflower very well while 72 (6.7%) had never heard of it. Some participants had used safflower infusions to treat anxiety and depression; 446 (44.4%) participants had never used it, but the remaining 558 (55.6%) had used it to varying degrees to treat anxiety and depression. Among the 752 participants who previously tried safflower, 279 (37.1%) reported that safflower was very effective, 389 (51.73%) reported some improvement, and 93 (12.36%) reported no improvement.

Conclusion

Emerging medical evidence is guiding herbal treatments. This research illustrates that more than 75% of the Saudi population are using Safflower to treat psychological stress. It elaborates that more than half of the population are already using safflower off the label to treat depression and anxiety and that they find it useful. A well-constructed clinical trial is thus critical to prove the evidence-based benefits of safflower in treating depression and anxiety. More studies on possible side effects are required to guarantee its safety. Nature has previously provided remarkable remedies, and more work will illustrate the value of safflower.

## Introduction

Rationale

“An herb is a friend of the physicians and a praise of the cooks.” - Charlemagne

Natural products can boost health in humans and animals, and they have a significant role in the prevention of diseases. These natural products have various biological properties such as antioxidant, anti-inflammatory, and anti-apoptotic activities. In vitro and in vivo studies have further established the usefulness of natural products in various pre-clinical models of neurodegenerative disorders [1].

In Arabic countries, funerals involve prayers at the mosque and tradition suggests that a safflower drink be included to soothe the mourners. Similarly, safflower is given in the puerperium period after delivery or even a miscarriage. Women are encouraged to add safflower to their drinks to help them cope with postpartum symptoms.

One Saudi study evaluated the prevalence, knowledge, and attitudes toward herbal medications used by Saudi women in the central region during pregnancy, labor, and after delivery. Of the 612 participants, 25.3%, 33.7%, and 48.9% used herbs during pregnancy, during labor, and after delivery, respectively. The primary motives for using herbal medicine during pregnancy, during labor, and after delivery were to boost general health, ease and accelerate labor, and clean the womb, respectively [2].

The safflower drink consists of safflower petals soaked in water until the water becomes yellow and the safflower aroma can be smelled and tasted. Although this traditional herbal recipe is easy, it is not broadly studied beyond local tradition. This review is targeted at physicians and pharmacists and the value it has for their patients, specifically psychiatric patients with depression and anxiety.

What is safflower?

Safflower (“Usfer”عصفر in Arabic and “Kafesheh” in Persian, anciently named “bastard saffron”) is a highly branched, herbaceous, thistle-like annual plant with many long sharp spines on the leaves. The plants are 30 to 150 cm tall with globular flower heads (capitula) and brilliant yellow, orange, or red flowers in July. Each branch will usually have from one to five flower heads containing 15 to 20 seeds per head [3].

Traditionally, the crop was grown for its flowers, used as a food additive, for making dyes, and in medicines. In the last 50 years, it has been cultivated mainly for the vegetable oil extracted from its seeds. Safflower oil is flavorless and colorless, and nutritionally similar to sunflower oil. It is used mainly as cooking oil, in salad dressing, and in the production of margarine. It may also be taken as a nutritional supplement. The International Nomenclature of Cosmetic Ingredients (INCI) identifier of safflower is *Carthamus tinctorius* [3].

## Materials and methods

A search of MEDLINE (PubMed), PsycINFO, Google Scholar, and Cochrane Library databases was conducted (up to September 19, 2021) on the use of safflower as herbal medicine. Several in vitro and in vivo clinical trials provide preliminary positive evidence for its antidepressant effects and anxiolytic activity. To date, however, there is no comprehensive review of safflower as an herbal antidepressant and anxiolytic with details on its psychopharmacology and applications in depression and anxiety in humans.

This research is a review and qualitative research. An electronic survey was done on Google Forms and distributed among the Saudi population through social media, thus assessing their knowledge about using safflower in treating depression and anxiety. The survey was distributed in Saudi Arabia in December 2021 and the results were finalized in January 2022.

Statistical analysis

Data analysis was performed using Statistical Package for the Social Sciences (SPSS) version 23 (IBM Corp., Armonk, NY). The frequency and percentages were used to display categorical variables. A chi-square test was used to test the association between categorical variables. The level of significance was set to 0.05.

Ethical approval

This research has been ethically approved by the Central Research Ethics Committee at Prince Sultan Military Medical City in Riyadh on December 22, 2021, as project number 2021-51.

## Results

A total of 1074 participants were included in the study. Table 1 shows the sociodemographic and academic profiles of the participants. As for the age, 15 (1.4%) participants were less than 18 years old, 44 (4.1%) were between 18 and 25 years, 176 (16.4%) were between 26 and 35 years, 340 (31.7%) were between 36 and 45 years, 297 (27.7%) were between 46 and 55 years, 168 (15.6%) were between 56 and 65 years, and 34 (3.2%) were older than 65 years. Of the participants, 100 (9.3%) were males and 974 (90.7%) were females. As for the education level, 61 (5.7%) participants had an education of less than a high school degree, 168 (15.6%) had a high school degree or equivalent, 102 (9.5%) had a college education but not a degree, 104 (9.7%) had an associate degree, 555 (51.7%) had a bachelor’s degree, 64 (6%) had a graduate degree, and 20 (1.9%) did not specify their education.

**Table 1:** Socio-demographic and academic profile of the participants (n = 1074).

Demographical characteristics		n	%
Age			
Less than 18 years		15	1.40
18-25 years		44	4.10
26-35 years		176	16.40
36-45 years		340	31.70
46-55 years		297	27.70
56-65 years		168	15.60
Older than 65 years		34	3.20
Gender			
Male		100	9.30
Female		974	90.70
Education level			
Less than high school degree		61	5.70
High school degree or equivalent		168	15.60
College but no degree		102	9.50
Associate degree		104	9.70
Bachelor’s degree		555	51.70
Graduate degree		64	6.00
Unspecified		20	1.90

Figure 1 displays the participants' previous knowledge of safflower. A total of 1002 (93.3%) participants reported they know safflower very well, while 72 (6.7%) reported they have never heard of it.

**Figure 1:** Participants' previous knowledge of safflower.

Figure 2 present the participants' source of information regarding safflower in participants who reported previously knowing safflower. A total of 775 (77.2%) participants reported they learned about safflower from family, 297 (29.6%) from social media, 214 (21.3%) from friends, 116 (11.6%) from books/publications, and 30 (3%) from other sources.

**Figure 2:** Participants' source of information regarding safflower.

Table 2 demonstrates the participants' thoughts regarding the therapeutic benefits of safflower and their previous experience with it. As for the participants' awareness of the therapeutic benefits of safflower, 178 (17.7%) participants reported that the safflower has some general medical uses, while 826 (82.3%) reported that they are aware that it is used in treating psychological stress. As for participants' use of safflower infusion for medical purposes in general, 282 (28.1%) participants reported they never used it, while the remaining 722 (71.9%) had a varying degree of using it for general medical purposes. As for participants' use of safflower infusion to treat psychological stress, 245 (24.4%) reported they never used it, while the remaining 759 (75.6%) had a varying degree of using it to treat psychological stress. As for participants' use of safflower infusion to treat anxiety and depression symptoms, 446 (44.4%) reported they never used it, while the remaining 558 (55.6%) had a varying degree to treat anxiety and symptoms of depression.

**Table 2:** Participants' thoughts regarding the therapeutic benefits of safflower and their previous experience with it (n = 1004).

Question	n	%
Q1. What are the therapeutic benefits of safflower that you are aware of?		
I know that it has general medical uses	178	17.7
Used in treating psychological stress	826	82.3
Q2. How often do you use safflower infusion for medical purposes in general?		
Always	59	5.9
Often	74	7.4
Sometimes	589	58.7
Never	282	28.1
Q3. How often do you use safflower infusion to treat psychological stress?		
Always	176	17.5
Often	135	13.4
Sometimes	448	44.6
Never	245	24.4
Q4. How often do you use safflower infusion to treat anxiety and depression symptoms?		
Always	92	9.20
Often	96	9.60
Sometimes	370	36.90
Never	446	44.40

Figure 3 illustrates the participants' reports on the improvement they experienced after using safflower. Among the 752 who previously tried safflower, 279 (37.1%) reported safflower was very effective, 389 (51.73%) reported they experienced some improvement, and 93 (12.36%) reported they experienced no improvement.

**Figure 3:** Participants' reports on the improvement they experienced after using safflower.

Figure 4 shows the participants' responses toward "Do you think safflower can be an effective medical treatment for symptoms of depression and anxiety?”. Of the participants, 834 (83.1%) reported that they think safflower can be effective in treating symptoms of depression and anxiety, while 170 (16.9%) did not think so.

**Figure 4:** Participants' responses toward "Do you think safflower can be an effective medical treatment for symptoms of depression and anxiety?”.

Table 3 displays the factors associated with previous knowledge of safflower. Age was significantly associated with previously knowing about safflower (p < 0.001). The highest rate of knowing about safflower was seen in those between 46 and 55 years (97.3%) and those between 36 and 45 (94.7), while the lowest rate was found in those younger than 18 years (73.3%), and those older than 65 years (85.3). Gender was also significantly associated with previously knowing about safflower (p < 0.001). Females had a notably higher rate of knowing about safflower compared to males (95.8% vs. 69%). Education level was also significantly associated with previously knowing about safflower (p < 0.001). The lowest rate of previously knowing about safflower was found in those with education less than high school (69.7%), while the highest rate of previously knowing about safflower was found in those with bachelor’s degrees (95.9%).

**Table 3:** Factors associated with previous knowledge of safflower. * Significant at level 0.05.

Factor	Previous knowledge of safflower		P-value
	Know it	Never heard of it	
Age			<0.001*
Less than 18 years	11 (73.3%)	4 (26.7%)	
18-25 years	40 (90.9%)	4 (9.1%)	
26-35 years	158 (89.8%)	18 (10.2%)	
36-45 years	322 (94.7%)	18 (5.3%)	
46-55 years	289 (97.3%)	8 (2.7%)	
56-65 years	153 (91.1%)	15 (8.9%)	
Older than 65 years	29 (85.3%)	5 (14.7%)	
Gender			<0.001*
Male	69 (69%)	31 (31%)	
Female	933 (95.8%)	41 (4.2%)	
Education level			<0.001*
Less than high school degree	59 (69.7%)	2 (3.3%)	
High school degree or equivalent	158 (94%)	10 (6%)	
College but no degree	93 (91.2%)	9 (8.8%)	
Associate degree	86 (82.7%)	18 (17.3%)	
Bachelor’s degree	532 (95.9%)	23 (4.1%)	
Graduate degree	57 (89.1%)	7 (10.9%)	

## Discussion

Safflower has been used for its therapeutic value for centuries. Ancient writings like “*Historia Plantarum,*” a botany book by John Ray published in 1686, mentioned the use of safflower in treating respiratory and gastrointestinal diseases.

The modern literature has numerous studies proving that safflower has therapeutic advances in multiple medical conditions [4]. On top of the list of the medicinal uses of safflower is its miraculous healing properties [5]. It can help the body heal via its anti-inflammatory mechanisms [6]. Safflower also has value in cardiovascular diseases [7], specifically ischemic conditions [8]. It can reverse cell death and regenerate adequate revascularization by angiogenesis [9].

Safflower can also overcome motor deficiencies in the central nervous system [10,11]. The natural compound hydroxysafflor yellow A (HSYA) isolated from the flower of the *Carthamus tinctorius* (safflower plant) can reduce apoptosis, partially pointing to the fact that HSYA protects against cerebral ischemia/reperfusion injury [12]. Hydroxysafflor yellow B (HSYB) has shown neuroprotective actions by recuperating the energy metabolism, scavenging free radicals, and decreasing lipid peroxides in the brain tissue [13]. Both compounds offer protection in response to cerebral ischemic reperfusion injury [14].

The flavonoid extract of safflower appears to have neuroprotective effects against neurotoxin-induced cellular and animal models of Parkinson’s disease [15]. Safflower has been included in the synthesis of NeuroAiD, a treatment used to support functional recovery after stroke [16]. It is also a complementary treatment for other brain injuries and Alzheimer's disease [17]. HSYA has been used to treat cardiovascular and cerebrovascular diseases clinically in China, but the drug target is still not clear [4].

Safflower (*Carthamus tinctorius*) has been used in food and traditional medicine due to its active compounds such as flavonoids, phenylethanoid glycosides, coumarins, fatty acids, and steroids to treat conditions such as dysmenorrhea, amenorrhea, and other diseases [18].

Using safflower in mental health

Lack of Research

The evidence for the efficacy of many complementary and alternative interventions used to treat anxiety and depression remains poor. Recent systematic reviews point to a significant lack of methodologically rigorous studies within the field. However, this lack of evidence does not diminish the popularity of such interventions within the general Western population [19].

Bipolar patients experience residual anxiety and insomnia between mood episodes and increasingly self-prescribe alternative medicines. Prior work concluded that adjunctive herbal medicines may alleviate these symptoms and improve outcomes in standard treatment despite limited evidence. Physicians need to have a more in-depth understanding of the evidence-based benefits, risks, and drug interactions of alternative treatments [20]. Even for alcoholism, the historical use of plant extracts to create herbal preparations for alcohol use treatment has been recorded, but their efficacy remains debatable, as further research is necessary [21].

A 2017 study showed that components (especially N-hexadecanoic acid) of *Carthamus tinctorius* extract induce antidepressant-like effects by interaction with dopaminergic (D1 and D2) and serotonergic (5HT1A and 5-HT2A receptors) systems. These findings validate the folk use of *Carthamus tinctorius* extract for the management of depression [22].

The most recent publication on safflower in treating mental illness was from Saudi Arabia earlier this year and it investigated Saudis' attitudes toward mental distress and psychotropic medications, attribution of causes, and expected side effects. This work analyzed participants' expectations toward alternative or complementary medicines using aromatic and medicinal plants via a survey. Here, 39 plants and herbs were reported by the participants and were a good start for creating a local library of medicinal plants traditionally used for treating mental distress. Mint (*Mentha sp.*) was the most commonly cited plant; it was mentioned 32 times. This was followed by chamomile (*Chamaemelum* *nobile*), suggested 22 times, anise (*Pimpinella anisum*), suggested 16 times, and lavender (*Lavandula sp.*) and safflower (*Carthamus tinctorius*), suggested 11 times each. Most of the reported plants and herbs have been documented for their psychological properties such as neuroprotective, anxiolytic, antidepressant, and anti-stress features via the inherent phytochemicals and secondary metabolites [23]. Surprisingly, only 18.8% of the participants agreed that medicinal and aromatic plants could treat psychological disorders. Participants (82%) reported that physicians are the most trustful and preferred source of information about alternative and complementary medicine [23].

Safflower (*Carthamus tinctorius*) petal extract exerts neuroprotective and antioxidant activities [24], which helps with its antidepressant and antianxiety properties [25]. A recent study was performed to evaluate the antianxiety and antidepressant effect of *Carthamus tinctorius* petal extract. The results show that *Carthamus tinctorius* produced very significant anxiolytic and antidepressant effects compared to control, similar to the standard anxiolytic and antidepressant drugs diazepam and nortriptyline. Hence, they concluded that safflower may be an alternative therapeutic while treating patients with anxiety and depressive disorders [25].

Lack of Human Studies

Safflower has been used in several cultures as a medicine for multiple conditions, especially mental illnesses, but such use is rarely recorded. No official clinical trial has yet measured its efficacy in treating mental illness in humans. This lack of human studies underscores the need to explore new treatments. Such a study is more feasible in some countries than others due to cultural beliefs and rituals.

Herbal teas with numerous ingredients, especially flowers, are common in traditional medicines and pharmacopeias of Greece and the Eastern Mediterranean. A study of traditional herbal mixtures with flowers shows their botanical ingredients and records the local medicinal uses of these mixtures in Greece, Lebanon, Syria, Iran, and Turkey. These mixtures are not consumed as a treatment when one is sick but rather to avoid getting sick as a preventive measure. The formulations can reach 40 ingredients (*Zhourat* in Arabic). The ingredients are usually whole or coarsely chopped in more traditional formulations, thus leading to the extreme variability of individual doses [26].

## Conclusions

Emerging medical evidence is guiding herbal treatments. This research illustrates that more than 75% of the Saudi population are using Safflower to treat psychological stress. It elaborates that more than half of the population are already using safflower off the label to treat depression and anxiety and that they find it useful. A well-constructed clinical trial is thus critical to prove the evidence-based benefits of safflower in treating depression and anxiety. More studies on possible side effects are required to guarantee its safety. Nature has previously provided remarkable remedies, and more work will illustrate the value of safflower.
